The article "Role of CD4+T, CD8+T Cells, and CD4+T/CD8+T Cell Ratio in Gastric Cancer and Its Clinical Significance" was retracted in 2023. Reasons: signs of a paper mill; suspected computer-generated content; unreliable results or conclusions; concerns about the data.

# Role of CD4^+^T, CD8^+^T Cells, and CD4^+^T/CD8^+^T Cell Ratio in Gastric Cancer and Its Clinical Significance

**DOI:** 10.1155/2022/1094607

**Published:** 2022-04-30

**Authors:** Jingqi Han, Linglin Zhao, Jianying Wu, Yinzhuo Diao, Qijing Guo, Jie Yang, Yushuang Luo

**Affiliations:** ^1^Department of Pathology, Affiliated Hospital of Qinghai University, Xining, China; ^2^Research Center for High Altitude Medicine, Qinghai University, Xining, China; ^3^Department of Emergency, Qinghai Provincial People's Hospital, Xining, China; ^4^Department of Virology, Qinghai Center for Disease Prevention and Control, Xining, China; ^5^Department of Oncology, Qinghai Province Cancer Hospital, Xining, China; ^6^Department of Oncology, Affiliated Hospital of Qinghai University, Xining, China

## Abstract

**Objective:**

To study the expression and clinical importance of CD4^+^T, CD8^+^T cells, and CD4^+^T/CD8^+^T cell percentage in gastric cancer (GC) patients.

**Methods:**

The blood count of CD4^+^T and CD8^+^T lymphocytes was ascertained via flow cytometry before surgery in 93 GC patients undergoing gastrectomy. The CD4^+^T, CD8^+^T, and Foxp3^+^T lymphocytes in cancerous and normal adjacent tissues and the presence of PD-L1 in cancerous tissues were detected via immunohistochemistry. The link between the permeation of CD4^+^T, CD8^+^T lymphocytes in venous blood, and cancer and normal adjacent tissues was analyzed.

**Results:**

Lauren histotype, TNM stage, lymphatic/nervous invasion, and NLR level were all considerably associated with peripheral CD4^+^T and CD8^+^T cell levels, whereas CD8^+^T lymphocytes were also associated with vascular invasion (*p* < 0.05). The CD4^+^T lymphocyte counts, CD4^+^T, and CD8^+^T cell percentage in GC tissues were found to have been decreased when compared to normal adjacent tissues, whereas the CD8^+^T and Foxp3^+^T lymphocyte count was higher in GC tissues (*p* < 0.05). According to a Spearman analysis, the CD4^+^T and CD8^+^T cell counts in tumor tissues were positively related to the Foxp3^+^T lymphocyte count (*p* < 0.05). Greater peripheral CD4^+^T lymphocyte counts and increased level of CD4^+^T/CD8^+^T percentage corresponded with greater CD4^+^T cell levels and increased CD4^+^T/CD8^+^T quantity in normal adjacent tissues. Higher levels of peripheral CD8^+^T cells corresponded with higher quantities of CD8^+^T cells in cancer tissues. A reduced CD4^+^T lymphocyte count, together with a reduced CD4^+^T/CD8^+^T percentage in venous blood, was consistent with a diminished CD4^+^T cell count along with a reduced CD4^+^T/CD8^+^T lymphocyte ratio in cancer and normal adjacent tissues.

**Conclusion:**

The peripheral quantity of CD4^+^T and CD8^+^T lymphocytes in GC patients can partly reflect the infiltrating state of these lymphocytes in cancer and normal adjacent tissues and can preliminarily predict immunotherapy response to a certain extent.

The article "Role of CD4+T, CD8+T Cells, and CD4+T/CD8+T Cell Ratio in Gastric Cancer and Its Clinical Significance" was retracted in 2023. Reasons: signs of a paper mill; suspected computer-generated content; unreliable results or conclusions; concerns about the data.

## 1. Introduction

Gastric cancer (GC) accounts for high incidence and mortality worldwide and is the fourth leading cause of cancer-related death globally, especially in Asian countries [1]. In recent years, it has been found that the occurrence and progression of malignant tumors are strongly correlated with the immune state of the body [2]. Simultaneously, high amounts of immunosuppressive factors are generated or secreted during the growth of tumors, which changes the immune microenvironment of the body and leads to eluding of tumor cells from immunosurveillance in the early stage [3]. Researches have indicated that T lymphocyte-mediated cytoimmunity plays a major role in the mechanism of antitumor immunity [4]. T lymphocytes are mainly divided into different functional subsets: helper (CD3^+^CD4^+^) T cells, killer (CD3^+^CD8^+^) T cells, regulatory T (Treg) cells, etc. CD8^+^T cells are the main antitumor effector cells, and CD4^+^T cells promote their activation and proliferation and the two synergistic antitumor, while Treg cells can induce tumor immunosuppression and immune escape [5]. The number and function of T lymphocyte subsets are abnormal in patients with malignant tumors, which leads to immune dysfunction and promotes tumor development [6].

At present, immunotherapy has a decisive and crucial contribution for the clinical treatment of cancer. In particular, the use of targeted immune inhibitors against the PD-L1 (programmed cell death-ligand 1) and/or PD-1 (programmed cell death 1) has ushered in a new era of cancer treatment via immune therapy. Although anti-PD-1 or anti-PD-L1 antibodies have been confirmed to excellent validity in many malignancies [7], yet in the nonscreening case, the response rate of monotherapy is only about 20% [8]. The infiltration of T lymphocytes and other immune cells in tumor microenvironment is a key factor affecting the efficacy of tumor immunotherapy [9]. Researches show that monitoring the changes of T lymphocyte subsets in tumor patients is of note to timely reflect the immune function and prognosis determination and observe the curative effect of tumor patients [10, 11]. Due to the complexity of tumor immunity, it is hard to comprehensively assess the tumor patients' immune status. Currently, the evaluation of the local tumor immune microenvironment is based on tumor tissue samples. However, various issues in actual clinical work make it difficult to obtain samples, and so the infiltration of immune cells in tumor tissues cannot be fully reflected. Hence, this study intends to observe and analyze the infiltration and relationship of CD4^+^T and CD8^+^T lymphocytes in peripheral venous blood and cancer tissues, in addition to the normal adjacent tissues of patients suffering from gastric cancer, to present theoretical support for the exploration of the method of evaluating the state of the tumor immune microenvironment and preliminary screening.

The article "Role of CD4+T, CD8+T Cells, and CD4+T/CD8+T Cell Ratio in Gastric Cancer and Its Clinical Significance" was retracted in 2023. Reasons: signs of a paper mill; suspected computer-generated content; unreliable results or conclusions; concerns about the data.

## 2. Methods

### 2.1. Specimen Source and Clinical Data

This was an observational prospective study. Cancer and matched normal adjacent tissue (5 cm away from the carcinoma border) samples were obtained from 93 GC patients undergoing gastrectomy in Qinghai University Affiliated Hospital from August 2019 to October 2021. The samples (4~5 *μ*m thick) were embedded in paraffin and sectioned. The seven inclusion criteria for patients were as follows: ① GC patients were diagnosed by pathological biopsy, without antitumor treatment prior to biopsy; ② the age ranged from 18 to 75 years; ③ the patients did not receive chemoradiotherapy and immunotherapy before the operation; ④ no other tumor was found; ⑤ there were no infections or autoimmune diseases in the preceding six months; ⑥ there was no serious organ dysfunction; ⑦ complete clinicopathological data and follow-up data were obtained. The clinical characteristics of 93 patients with GC included were described in columns 1 and 2 of Table 1. The patients chosen belonged to the age group of 35-75 years (mean, 56.44 ± 8.25 years). Then, the average age was 56 years. Table 1 details the baseline clinical description of 78 patients (83.9%) had an ECOG score (Eastern Cooperative Oncology Group performance status) of patients 0-1. All patients with stage IV gastric cancer enrolled in this study were patients without distant metastasis (T1-3N3M0 and T4N2M0). Prior approval from the ethical committees of Qinghai University allied hospital (No.: SL-20190014) was obtained for the conduct of this clinical research and was examined thoroughly. Each recruited patient involved in this study voluntarily signed the informed consent forms.

### 2.2. Reagents and Instruments

Erythrocyte lysate, EDTA-K2 antigen repair solution, PBS phosphate buffer, rabbit anti-human CD4, CD8, Foxp3 monoclonal antibody, immunohistochemical Ultrasensitive™ SP detection kit, DAB color detection kit, and Ventana PD-L1 (SP263) kits were purchased from Fuzhou Mai Xin Biotechnology Development Co., Ltd; BD Multitest™ CD45/CD3/CD4/CD8/Monoclonal Antibody and BD Trucount™ Tubes were purchased from BD Bioscience (USA). Flow cytometry (FCM) analyses (FACS Calibur, BD) and immunohistochemistry autostainer (Roche Benchmark XT Roche) were employed.

The article "Role of CD4+T, CD8+T Cells, and CD4+T/CD8+T Cell Ratio in Gastric Cancer and Its Clinical Significance" was retracted in 2023. Reasons: signs of a paper mill; suspected computer-generated content; unreliable results or conclusions; concerns about the data.

### 2.3. Flow Cytometry

Venous blood samples of 2 ml were collected from 93 GC patients who met the above inclusion criteria one day before gastrectomy and added into an EDTA-K2 anticoagulant tube. Each blood sample (50 *μ*l) was added into BD Trucount™ Tubes, then the following antibodies were added to each tube: CD3-FITC, CD45-PerCP, CD4-APC, and CD8-PE, and the procedure was conducted according instruction manual. The entire count of CD3^+^CD4^+^T plus CD3^+^CD8^+^T cell in surrounding venous blood was measured by FCM and analyzed via the MultiSET automatic software (Figure 1) and recorded as cell count/*μ*l.

### 2.4. Pathology and Immunohistochemistry (IHC)

The CD4^+^, CD8^+^T lymphocytes, and Treg (Foxp3^+^) cells in carcinoma and normal adjacent units were detected using an SP immunohistochemical staining kit, and PD-L1 expression was detected by using Ventana PD-L1 (SP263) assay. Five areas with the most abundant lymphocyte infiltration were selected in the low-power microscopic field (×100), then the positively stained cells were counted under high magnification (×400), and the mean percentage of the five fields was expressed as CD8^+^T cells, cells/HPF CD4^+^, and Tregs (Foxp3^+^) in carcinoma and normal adjacent tissues (Figure 2). PD-L1 positive cells in cancer tissues are shown in Figure 3. PD-L1 positive was defined as CPS ≥ 10%, and PD-L1 negative was CPS < 10% [12]. Each slice was examined by two pathologists using a double-blind method.

### 2.5. Statistical Analysis

The software used for statistical analysis and mapping were the SPSS 25.0 and GraphPad Prism 8.3. The normality test for the measurement data was all skewness data, expressed by median and quartile M (P25 and P75). For comparison between the two groups, the Wilcoxon test was carried out for analyzing the combined data, Mann-Whitney *U*-test was used for analyzing the separated data. To analyze the multiple groups, the test of Kruskal-Wallis was utilized. The correlation coefficient was calculated by the Spearman rank test. *p* < 0.05 was considered as the indicator for statistical difference, and the *p* values were bilateral.

## 3. Results

### 3.1. Relationship between the Number and Ratio of CD4^+^T, CD8^+^T Cells in the Surrounding Blood, and Clinical Features in GC Patients

No crucial or appreciable relation was noted in the peripheral blood between the count of CD4^+^T cells with gender, age, tumor location, differentiation degree, histological type, vascular invasion, Ki67, and PLR (*p* > 0.05); it was directly related to Lauren type, TNM stage, lymph node/nerve invasion, and NLR level (*p* < 0.05). The levels of peripheral blood CD4^+^T cells of patients with TNM I-II stages and without lymph node and nerve invasion were higher. The amount of CD4^+^T lymphocytes in the surrounding blood was higher in Lauren intestinal-type patients when equated to mixed and diffuse-type patients. The peripheral blood CD8^+^T cell count was not significantly correlated with gender, age, tumor location, differentiation, histological type, Ki67, and PLR (*p* > 0.05) but was particularly associated with Lauren type, lymph node, TNM stage, nerve and vascular invasion, and NLR level (*p* < 0.05). The peripheral blood CD8^+^T cells of patients with TNM stages I-II, Lauren intestinal type, no lymph node, and neurovascular invasion were higher. The CD4^+^T and CD8^+^T cell count in the surrounding blood was inversely related to NLR. As detailed in Table 1, no correlation is observed between the ratio of CD4^+^T/CD8^+^T cell in the peripheral (surrounding) blood and the above clinical characteristics (*p* > 0.05, Table 1).

The article "Role of CD4+T, CD8+T Cells, and CD4+T/CD8+T Cell Ratio in Gastric Cancer and Its Clinical Significance" was retracted in 2023. Reasons: signs of a paper mill; suspected computer-generated content; unreliable results or conclusions; concerns about the data.

### 3.2. Distribution of CD8^+^T, CD4^+^T Lymphocytes, and Treg (Foxp3^+^) Cell in Cancerous and Normal Adjacent Tissues

Wilcoxon paired signed-rank test detailed in Table 2 was used for evaluating the results: CD4^+^T lymphocytes in GC tissues were decreased than in the neighboring tissues (median 55.90 vs. 70.50, *p* = 0.004); the CD4^+^T/CD8^+^T percentage in carcinoma tissues was lesser in contrast to the normal adjacent tissues (median 0.84 vs. 1.11, *p* = 0.001); CD8^+^T and Foxp3^+^T lymphocyte count was elevated in malignant tissues as compared to that of the normal adjacent tissues (median 72.90 vs. 65.60, *p* = 0.038) and (median 29.00 vs. 16.00, *p* < 0.001).

Positive correlation was demonstrated by the correlation analysis (Spearman's correlation analysis) between the CD4^+^T, CD8^+^T count, and Foxp3^+^T lymphocytes in tumor tissues (*p* < 0.05) (Figure 4).

### 3.3. Relationship between the Number of CD4^+^T Lymphocytes and CD8^+^T Lymphocytes in Peripheral Blood and Their Infiltration in Cancerous and Normal Adjacent Tissues

The following results can be observed in Table 3. When the peripheral levels of CD4^+^T lymphocytes were “high,” their levels in the normal adjacent tissues and cancer tissues were also high in 44 and 31 cases, respectively. Consistency between peripheral blood and normal adjacent tissues was 95.7% (44/46), higher than that between peripheral blood and cancer tissues 67.4% (31/46). When the peripheral CD8^+^T lymphocytes were “high,” their quantity in the normal adjacent tissues and cancer tissues was also high in 37 and 43 cases, respectively. Consistency between peripheral blood and cancer tissues was 100% (43/40), higher than that between peripheral blood and normal adjacent tissues 92.5% (37/40). When CD4^+^T/CD8^+^T proportion was “high” in the surrounding blood, the CD4^+^T and CD8^+^T cells measured in adjacent and cancer tissues were high as well in 37 and 22 cases, respectively. Consistency between peripheral blood and normal adjacent tissues was 78.7% (37/47), higher than that between peripheral blood and cancer tissues 46.8% (22/47). Consistent with diminished quantities of CD4^+^T and a lesser percentage of lymphocytes (CD4^+^T/CD8^+^T) in the peripheral blood, these parameters were also low in normal adjacent tissues and cancer tissues (49/47, 62/47 and 56/46, 71/46).

The article "Role of CD4+T, CD8+T Cells, and CD4+T/CD8+T Cell Ratio in Gastric Cancer and Its Clinical Significance" was retracted in 2023. Reasons: signs of a paper mill; suspected computer-generated content; unreliable results or conclusions; concerns about the data.

Combined with the presence of PD-L1 in gastric cancer cells, the CD4^+^T and the CD8^+^T quantities in cancer tissues and normal adjacent tissues of PD-L1 expressing patients were considerably greater than the negative counterparts of PD-L1 (*p* < 0.05) (Table 4).

## 4. Discussion

In the antitumor immunity dominated by cellular immunity, T lymphocyte subsets of distinct functions exert antitumor properties by modulating immune activity [13]. CD4^+^ protein moieties are present on the outer membrane of helper T cells (TH) and inducible T cells (Ti). CD8^+^ molecules are primarily expressed on the outer membrane of T cells with regulatory effect and cytotoxic T cells (TC) with killing effect [14]. Studies have shown that [15] in the process of malignant tumor formation, Soluble immunosuppressive factors secreted by cancerous cells could inhibit CD4^+^T cell proliferation and differentiation, whereas CD8^+^T cells dominated by TS have increased reactivity, which in turn has a modulatory or suppressive effect on CD4^+^T cells, leads to a reduction in CD4^+^/CD8^+^ ratio, and leaving the immune microenvironment toward an immunosuppressive state. Previous study detected that a lower peripheral blood CD4^+^/CD8^+^ ratio is associated with shorter OS and increased risk of death, which can be used as a prognostic indicator of OS [16]. The CD4^+^T and CD8^+^T lymphocyte counts in the peripheral blood of GC patients were found to be substantially correlated with Lauren classification, TNM stage, lymph node metastases, nerve invasion, and NLR level, with CD8^+^T lymphocytes also being related to vascular invasion in this investigation. The cell count of CD4^+^T and CD8^+^T was inversely proportional to the level of NLR in the surrounding blood. NLR is the ratio of neutrophils to lymphocytes in peripheral blood, reflecting the stability of inflammatory response and immune function in the body [17]. The number of CD4^+^T and CD8^+^T lymphocytes in the surrounding blood decreases with the increase of NLR, indicating the improvement of the inflammatory response and the reduction of antitumor immune function, thus leading to tumor recurrence and metastasis. Hence, detection of the number of CD4^+^T and CD8^+^T cells in peripheral blood combined with NLR and PLR has certain significance for assessing the condition and prognosis of GC subjects.

The article "Role of CD4+T, CD8+T Cells, and CD4+T/CD8+T Cell Ratio in Gastric Cancer and Its Clinical Significance" was retracted in 2023. Reasons: signs of a paper mill; suspected computer-generated content; unreliable results or conclusions; concerns about the data.

Hiraoka et al. [18] found that the degree of intrusion of CD8^+^T and CD4^+^T lymphocytes in the lung cancer stroma was increased than that in the tumor. A high ratio of CD4^+^ to CD8^+^T in ovarian cancer tissue predicts a good prognosis [19]. Immunohistochemical staining of the present study indicates that the CD4^+^T counts and CD4^+^T to CD8^+^T lymphocyte ratios in cancerous tissues of GC patients were notably reduced as to those in paracarcinoma tissues (*p* < 0.05). However, the CD8^+^T cell count was higher in GC tissues as to the paracarcinoma in this study, which is inconsistent with the relevant reports, and this difference is considered to be related to the immune subtypes with different responsibilities of CD8^+^T cells. Furthermore, our result shows that the amount of Foxp3^+^T cells in GC tissues was elevated than that of the adjacent normal tissues. Forkhead transcription factor P3 (Foxp3) is a key intracellular indicator for regulatory T cell [20]. Abundant evidence shows that Tregs contribute to immune evasion and tumor growth via encouraging the formation of immunosuppressive microenvironment, and its density is related to shorter OS [21, 22]. A study had found that [23] Foxp3 was expressed in CD8^+^CD28^−^T plus CD4^+^CD25^+^T cells and has a negative regulatory effect on immune function generated by T cell activation. In the current study, Spearman correlation analysis presents a positive connection between the distribution of CD4^+^T: Foxp3^+^T cells and CD8^+^T: Foxp3^+^T cells in cancer tissues (*p* < 0.05); however, there was no any considerable correlation in the normal adjacent tissues. This suggests that the increased CD8^+^T cells in cancerous cells may be induced CD8^+^Treg cells, which participate in immunosuppression and promote tumorigenesis and development. However, their types and functions need to be further studied.

Recent research indicates that [24] the effectiveness of immune checkpoint blockers is positively associated with the degree of T lymphocyte infiltration. Chen and Mellman [25] divided the tumor immune microenvironment into three types: immune-inflamed, immune desert-type, and immune excluded-type, by analyzing the immunohistochemical results of a large number of tumor specimens before treatment and combining these results with their overall reaction to PD-L1/PD-1 targeted inhibitors. We observed in the present research conducted that the elevated counts of CD4^+^T and CD8^+^T cells in peripheral blood were more consistent with CD4^+^T plus CD8^+^T cell numbers in normal adjacent tissues. We can boldly assume that the tumor immune phenotype may tend to be “immuno-inflammatory” or “immune-privileged”, if PD-L1 is positive, on the basis of immune checkpoint inhibitors, it promotes T cell migration to tumor tissue, transforming “cold tumors” into “hot tumors” is the key to improving anti-tumor therapy. When the peripheral blood CD4^+^T, CD8^+^T cell numbers, and the ratio of CD4^+^T to CD8^+^T in GC patients were all at low levels, the peripheral blood, carcinoma tissues, and paracarcinoma tissues were completely consistent and all had low cell counts. We can evaluate the lack of effector T cells in both the internal and peripheral environment of tumor cells by peripheral blood. In this case, the tumor immunophenotype may be the immune-desert phenotype, anti PD-1/PD-L1 therapy had little effect and poor prognosis. However, for a minority of PD-L1-positive patients, a variety of neoadjuvant therapies such as chemotherapy, radiation therapy, and oncolytic virotherapy can be performed in advance [26, 27] to improve the infiltration and function of effector cells in the tumor immune microenvironment, and then, treatment targeting immune checkpoints can be performed.

The article "Role of CD4+T, CD8+T Cells, and CD4+T/CD8+T Cell Ratio in Gastric Cancer and Its Clinical Significance" was retracted in 2023. Reasons: signs of a paper mill; suspected computer-generated content; unreliable results or conclusions; concerns about the data.

The lymphocyte subsets in tumor tissue more closely reflect the tumor microenvironment than those in peripheral blood [28]. However, it is not easy to acquire samples in clinical work or else the amount of tissue is insufficient to reflect the status of infiltrating lymphocytes in tumor tissue. The detection method using peripheral blood lymphocytes is simple, easy to repeat, and less traumatic. In this study, we found that it can indirectly assess the degree of intrusion of CD4^+^T and CD8^+^T in cancer and paracarcinoma tissues of GC patients via detecting the CD4^+^T and CD8^+^T cell numbers present in the surrounding blood, combined with the presence of PD-L1, and the immunotherapy response may be better predicted. However, this study still has some deficiencies and limitations. For instance, the normal reference values of CD4^+^T plus CD8^+^T cell numbers and CD4^+^T/CD8^+^T cell ratio in blood have no unified standard for the distinguished cut-off value due to vary races, economic conditions, and living environment [29, 30]. Prognosis analysis was not performed due to the lack of follow-up. peripheral blood Foxp3 T cell subtype was not detected in present study. As a consequence of the relatively small sample size and large heterogeneity of clinical samples in this study, further exploration and verification should be conducted in a wider range of clinical studies in the next step to determine the reliability of the study results and further refine molecular typing detection.

The article "Role of CD4+T, CD8+T Cells, and CD4+T/CD8+T Cell Ratio in Gastric Cancer and Its Clinical Significance" was retracted in 2023. Reasons: signs of a paper mill; suspected computer-generated content; unreliable results or conclusions; concerns about the data.

## Figures and Tables

**Figure 1:** Four-color flow cytometric plots of CD3^+^CD4^+^T cells and CD3^+^CD8^+^T cells in the peripheral blood.

**Figure 2:** Infiltration of CD4^+^T, CD8^+^T, and Foxp3^+^T cells in malignant tissues and normal adjacent tissues. CD4^+^T plus CD8^+^T cells were stained in yellow or brownish yellow on the cell membrane or cytoplasm, and the nuclear was brown or tan as Foxp3^+^T cells (×400), scale bar: 20 *μ*m.

**Figure 3:** Positive PD-L1 in GC cells and staining was located in the cell membrane or cytoplasm, showing brown-yellow particles, scale bar: 20 *μ*m.

**Figure 4:** (a, c) Spearman correlation analysis showed a positive correlation among the CD4^+^T cells and CD8+T cells with Foxp3^+^T cells in tumor tissues (*p* < 0.05); (b, d) no considerable or pronounced correlation was observed between CD4^+^T: Foxp3^+^T cells and CD8^+^T: Foxp3^+^T cells in normal adjacent tissues (*p* > 0.05).

**Table 1:** Relationship between the number of CD4^+^T and CD8^+^T cells in peripheral blood and clinicopathological features in GC patients (M (P25 and P75)).

Clinicopathological features	*n* (%)	CD4^+^T (cells/*μ*l)	*p*	CD8^+^T (cells/*μ*l)	*p*	CD4^+^T/CD8^+^T	*p*
Gender							
Male	63 (67.7)	553.00 (430.00, 668.00)	0.318	398.00 (301.00, 501.00)	0.322	1.28 (1.09,1.64)	0.115
Female	30 (32.3)	572.50 (448.00, 748.50)		387.50 (192.25, 487.25)		1.44 (1.15, 2.42)	
Age(years)							
<60	56 (60.2)	563.00 (340.25, 703.25)	0.461	397.50 (228.25, 514.75)	0.635	1.26 (1.12, 1.60)	0.197
≥60	37 (39.8)	560.00 (473.50, 676.00)		399.00 (301.50, 480.00)		1.36 (1.14, 2.33)	
Histological type							
Adenocarcinoma	74 (79.6)	572.50 (473.50, 727.75)	0.056	403.50 (304.25, 493.25)	0.446	1.33 (1.14, 1.75)	0.584
Signet-ring+mucinous adenocarcinoma	19 (20.4)	462.00 (364.00, 574.00)		327.00 (264.00, 623.00)		1.22 (0.98, 1.64)	
Pathological type							
Well differentiation	28 (30.1)	523.00 (330.5, 876.00)	0.927	387.50 (305.5, 525.25)	0.957	1.40 (1.14, 1.84)	0.773
Low differentiation	65 (69.9)	569.00 (448.00, 629.00)		399.00 (264.00, 490.00)		1.29 (1.13, 1.64)	
Lauren classification							
Intestinal type	40 (43.0)	635.50 (520.00, 828.25)	**<0.001**	452.50 (382.25, 544.75)	**0.007**	1.39 (1.23, 1.60)	0.091
Mixed type	24 (25.8)	561.00 (340.25, 664.50) ^**a**^		348.50 (241.00, 479.75)^a^		1.49 (1.08, 1.92)	
Diffuse type	29 (31.2)	448.00 (281.00, 562.50) ^**b**^		328.00 (195.00, 469.50)^b^		1.17 (0.78, 1.59)	
Tumor location							
Gastric cardia	34 (36.5)	572.50 (413.75, 650.25)	0.730	412.50 (233.00, 495.00)	0.669	1.39 (1.15, 1.75)	0.839
Gastric body	22 (23.7)	553.00 (458.50, 784.00)		395.50 (304.00, 609.75)		1.29 (1.14, 1.60)	
Gastric antrum	37 (39.8)	560.00 (428.50, 686.00)		398.00 (268.50, 485.50)		1.29 (1.00, 1.88)	
TNM stage							
I~II	45 (48.4)	637.00 (490.00, 818.50)	**0.001**	458.00 (327.50, 516.00)	**0.019**	1.40 (1.17, 1.81)	0.161
III~IV	48 (51.6)	494.00 (372.00, 577.00)		350.50 (211.00, 450.75)		1.26 (1.01, 1.64)	
Lymph node metastasis							
Absent	23 (24.7)	664.00 (553.00, 736.00)	**0.002**	488.00 (458.00, 558.00)	**<0.001**	1.26 (1.18, 1.59)	0.824
Present	70 (75.3)	506.50(359.75, 637.50)		365.50 (226.75,448.25)		1.33 (1.11, 1.90)	
Nerve invasion							
Absent	63 (67.8)	578.00 (487.00, 725.00)	**0.006**	399.00 (326.00, 515.00)	**0.042**	1.38 (1.14, 1.74)	0.435
Present	30(32.2)	472.00 (292.25, 585.50)		338.50 (193.00, 484.00)		1.22 (1.12, 1.71)	
Vascular invasion							
Absent	51 (54.8)	572.00 (483.00, 701.00)	0.214	438.00 (341.00, 555.00)	**0.012**	1.29 (1.12, 1.59)	0.316
Present	42 (45.2)	558.50 (334.75, 661.50)		364.00 (221.25, 475.50)		1.32 (1.14, 1.96)	
Ki67							
≤30%	34 (36.6)	607.50 (485.25, 701.75)	0.239	442.50 (338.00,554.25)	0.057	1.26 (1.11, 1.61)	0.225
>30%	59 (63.4)	529.00 (431.00, 694.00)		395.00 (227.00,473.00)		1.36 (1.14, 1.91)	
NLR							
High NLR	47 (50.5)	493.00 (308.00, 654.00)	**0.010**	341.00 (207.00, 462.00)	**0.009**	1.26 (0.78, 1.74)	0.298
Low NLR	46 (49.5)	586.00 (486.75, 709.25)		449.50 (348.75, 518.50)		1.34 (1.18, 1.67)	
PLR							
High PLR	47 (50.5)	557.00 (438.00, 668.00)	0.875	399.00 (227.00, 494.00)	0.684	1.33 (1.14, 1.74)	0.642
Low PLR	46 (49.5)	570.50 (436.75, 709.255)		398.00 (301.75, 498.25)		1.29 (1.05, 1.67)	

Note: NLR was peripheral blood neutrophil count/lymphocyte count; PLR was peripheral blood platelet count/lymphocyte count; taking the median NLR and PLR (1.96 vs. 117.24) as the cut-off value, 93 GC patients were categorized into high NLR group and low NLR group and high PLR group and low PLR group. Bold fonts are considered to have significant differences. ^a^Correlated with the intestinal type group *p* < 0.05; ^b^compared with the intestinal type group *p* < 0.01.

The article "Role of CD4+T, CD8+T Cells, and CD4+T/CD8+T Cell Ratio in Gastric Cancer and Its Clinical Significance" was retracted in 2023. Reasons: signs of a paper mill; suspected computer-generated content; unreliable results or conclusions; concerns about the data.

**Table 2:** Comparability of CD4^+^T, CD8^+^T, Foxp3^+^T cell count between carcinoma and normal adjacent tissues.

Group	*n*	CD4^+^T (cells/HPF)	CD8^+^T (cells/HPF)	Foxp3^+^T (cells/HPF)	CD4^+^T/CD8^+^T
Cancer tissues	93	55.90 (34.40, 90.70)	72.90 (43.03, 102.15)	29.00 (13.50, 53.07)	0.84 (0.51, 1.26)
Normal adjacent tissues	93	70.50 (48.90, 103.00)	65.60 (42.95, 94.20)	16.00 (9.00, 24.50)	1.11 (0.77, 1.63)
*Z*		2.881	2.071	5.895	3.418
*p*		**0.004**	**0.038**	**p** < 0.001	**0.001**

Results are expressed as median (P25 and P75). Bold fonts are considered to have significant differences.

**Table 3:** Relationship between the levels of CD4^+^T and CD8^+^T in the peripheral blood to that of the carcinoma and normal adjacent tissues.

Group	CD4^+^T		CD8^+^T		CD4^+^T/CD8^+^T	
	High	Low	High	Low	High	Low
Peripheral blood	46 (49.5)	47 (50.5)	40 (43.0)	53 (57.0)	47 (50.5)	46 (49.5)
Normal adjacent tissues	44 (47.3)	49 (52.7)	37 (39.8)	56 (60.2)	37 (39.8)	56 (60.2)
Cancer tissues	31 (33.3)	62 (66.7)	43 (46.2)	50 (53.8)	22 (23.7)	71 (76.3)

Note: The mean value of CD4^+^T and CD8^+^T in peripheral blood and tissues of 93 individuals was calculated as the cut-off value (high vs. low). CD4^+^T cells ≥ 565.10/*μ*l and CD8^+^T cells ≥ 421.55/*μ*l in peripheral blood, CD4^+^T cells ≥ 74.25/HPF and CD8^+^T cells ≥ 75.78/HPF in tissues were defined as “high”; CD4^+^T/CD8^+^T ratio ≥ 1.31 (the mean ratio was 1.31) was considered to be “high.” Results are presented as the number of cases (proportion).

**Table 4:** Connection between PD-L1 expression in cancerous cells and the cell count of CD4^+^T and CD8^+^T in peripheral blood, surrounding tissues, and cancer tissues.

M (P25 and P75)	PD-L1 expression		*Z*	*p*
	Positive *n* (%) 35 (37.6)	Negative *n* (%) 58 (62.4)		
Peripheral blood (cells/*μ*l)				
CD4^+^T	572.00 (483.00, 725.00)	521.00 (359.76, 657.50)	1.642	0.101
CD8^+^T	458.00 (341.00, 501.00)	390.50 (249.25, 476.50)	1.475	0.140
CD4^+^T/CD8^+^T	1.38 (1.15, 1.76)	1.28 (1.09, 1.67)	0.781	0.435
Normal adjacent tissues (cells/HPF)				
CD4^+^T	88.00 (49.40, 100.00)	67.15 (48.40, 107.10)	0.230	0.818
CD8^+^T	80.50 (50.30, 98.50)	59.20 (36.78, 85.51)	1.991	**0.047**
CD4^+^T/CD8^+^T	1.08 (0.67, 1.41)	1.15 (0.82, 2.05)	1.435	0.151
Cancer tissues (cells/HPF)				
CD4^+^T	70.00 (48.70, 115.60)	49.99 (26.79, 77.42)	2.657	**0.008**
CD8^+^T	90.70 (67.00, 127.50)	56.50 (35.80, 85.42)	3.799	**<0.001**
CD4^+^T/CD8^+^T	0.70 (0.45, 1.26)	0.90 (0.59, 1.27)	1.277	0.202

Results are expressed as median (P25 and P75). Bold fonts are considered to have significant differences.

## Data Availability

On reasonable request, the corresponding author can provide the dataset to the support findings of the current study.
